The article "Diffusion-Weighted Imaging Combined with Perfusion-Weighted Imaging under Segmentation Algorithm in the Diagnosis of Melanoma" was published in 2022. Journal: Contrast Media Mol Imaging.

# Diffusion-Weighted Imaging Combined with Perfusion-Weighted Imaging under Segmentation Algorithm in the Diagnosis of Melanoma

**DOI:** 10.1155/2022/1968189

**Published:** 2022-06-27

**Authors:** Chuankui Shi, Peng Ge, Yuping Zhao, Guobao Huang

**Affiliations:** ^1^Department of Dermatology, Qilu Children's Hospital of Shandong University, Jinan 250022, Shandong, China; ^2^Burn and Plastic Surgery, The People's Hospital of Zhangqiu Area, Zhangqiu Area, Jinan 250200, Shandong, China; ^3^Burn and Plastic Surgery, Central Hospital Affiliated to Shandong First Medical University, Jinan 250013, Shandong, China

## Abstract

This study is aimed at exploring the value of magnetic resonance diffusion-weighted imaging (DWI) combined with perfusion-weighted imaging (PWI) for diagnosing melanoma under a three-dimensional (3D) hybrid segmentation algorithm. 40 patients with melanoma were collected as research objects and subjected to magnetic resonance imaging (MRI) examination. A segmentation model was constructed and the original images were input. The noise contained in the images was preprocessed and normalized, and the mixed level set segmentation was performed after linear fusion of the images. Imaging findings were analyzed to find that the combined diagnosis of DWI and PWI with a 3D hybrid segmentation algorithm had the advantage of being clear and accurate. 10 primary cases were detected, which occurred in the cerebral meninges; 30 cases of metastases occurred inside the skull, mostly adjacent to the surface of the brain. The typical T1-weighted imaging (T1WI) and T2-weighted imaging (T2WI) of melanoma showed high signal and low signal, respectively, and the enhanced scan showed obvious enhancement. Atypical melanoma was manifested variously in MRI; a few had cystic necrosis, and an enhanced scan of the solid area revealed significant enhancement. Patients with multiple metastatic melanomas mainly showed low signal on DWI, and patients with primary or single metastatic melanoma mainly showed high signal or mixed high signal. Patients with perfusion imaging showed high perfusion on PWI. The 3D hybrid segmentation algorithm helped to improve the accuracy of DWI combined with PWI in the diagnosis of melanoma. This work provided a certain reference for the clinical diagnosis of melanoma.

## 1. Introduction

Melanoma generally refers to malignant melanoma in clinical practice, which is a kind of malignant tumor derived from melanocytes. Its pathogenesis is not yet clear. Relevant studies indicate that its occurrence and development are closely related to the genes, the environment, or the genes together with the environment. The occurrence of this disease is relatively insidious, and the prognosis of patients is poor [1]. Malignant melanoma is more common in adults over 30 years old and is slightly less in men than women. It usually occurs in skin, mucous membranes, and organs, but it can also occurs in the eyes, nasal cavity, and the brain sometimes. It can be newly caused by dysplastic nevus, and the malignant transformation of junctional nevus and congenital or acquired benign melanocytic nevus, accounting for about 3% of all tumors [2, 3]. Signs of malignant transformation are generally manifested as the increase of the pigment volume, the darkening of the color, the sudden growth, and the appearance of inflammation, ulcers, and bleeding of the nevus [4]. In recent years, the incidence and mortality of malignant melanoma have increased gradually, and the age of death is even smaller than that of other solid tumors. Early clinical diagnosis of some melanomas is relatively difficult, and puncture or biopsy is not recommended [5].

The article "Diffusion-Weighted Imaging Combined with Perfusion-Weighted Imaging under Segmentation Algorithm in the Diagnosis of Melanoma" was published in 2022. Journal: Contrast Media Mol Imaging.

Histopathological examination is the gold standard for diagnosing melanoma, and imaging examinations can accurately locate and quantitatively analyze the lesions. These are helpful for the selection of treatment plans, prediction of therapeutic effect, and follow-up in the latter period, having clinical significance. Computed tomography is a common imaging method in clinical practice. However, some patients think that it is not sensitive to early limited-stage metastases of melanoma, has a low benefit rate, and cannot display limbs and other body parts. Conventional magnetic resonance imaging (MRI) gives a better resolution for soft tissues without radiation and can analyze the tissue source and signal characteristics of lesions on purpose, which is of great value in diagnosing melanoma [6, 7]. It can obtain information such as blood flow, metabolism, and biochemistry and display microscopic images and data noninvasively. Thus, the diagnosis of cancer can be focused on microscopic changes rather than morphology, and the biological characteristics of cancer tissues can be better displayed. It also makes the detailed information of the cancer tissues fully known, and the diagnosis rate and treatment rate can be improved [8, 9]. Diffusion-weighted imaging (DWI) and perfusion-weighted imaging (PWI) have fully demonstrated their application value and potential in the brain, liver, and prostate cancers. It was suggested that they could be used for the differentiation of benign and malignant cancers, the monitoring of postoperative recurrence, and the efficacy analysis of radiotherapy and chemotherapy, etc. [10]. DWI is an ideal method to detect the diffusion movement of water molecules in living tissues by using diffusion-sensitive gradients. An apparent diffusion coefficient is a physical quantity of the diffusion ability of water molecules that is used to quantitatively describe the diffusion movement of water molecules in the tissues [11]. PWI appeared with the rapid imaging sequence of MRI. It is an imaging technique that noninvasively evaluates the blood perfusion of the tissues by observing and comparing the early characteristics of tissue distribution [12].

The article "Diffusion-Weighted Imaging Combined with Perfusion-Weighted Imaging under Segmentation Algorithm in the Diagnosis of Melanoma" was published in 2022. Journal: Contrast Media Mol Imaging.

In image processing, there are countless algorithms that can be applied for segmentation. The earliest method used for automatic segmentation of cerebral tumor is traditional machine learning, in which the threshold algorithm, clustering algorithm, and deformation mode algorithm are more commonly used than other machine learning algorithms [13, 14]. Automatic brain tumor segmentation technology has been a hot research topic in recent years, especially that based on multimodal three-dimensional (3D) image segmentation. The high precision and low deviation of the segmentation method have become common goals in surgical plans [15]. The technology can meet the needs of clinical medical treatment and has high segmentation accuracy and research prospects [16, 17]. However, many existing methods around the world are on the basis of a single modality, so their segmentation accuracy and reliability are not very high. Thus, the 3D hybrid segmentation algorithm was innovatively applied to DWI and PWI, and the diagnostic data of intracranial melanoma were expounded. This provided a theoretical basis for further understanding of melanoma and improved the accuracy of clinical diagnosis.

## 2. Materials and Methods

### 2.1. General Data

In this study, 40 patients with central nervous melanoma were included, and they were admitted to hospital from September 2019 to September 2020. All the patients, including 30 males and 10 females, were 37–68 years old with an average age of 44.35 ± 9.78. At the time of visiting doctor, patients with symptoms like nausea, vomiting, dizziness, headache, weakness of the limbs, visual disturbances, and confusion of consciousness had lesions in the brain. Meanwhile, the patients with stiff necks accompanied by soreness had lesions in the spinal canal. The informed consents were signed by the patients and their families. This study has been approved by the ethics committee of the hospital.

The inclusion criteria were as follows: patients were diagnosed clearly by histopathological examination; Patients had the complete clinical and pathological data; Patients had a good physical condition generally. The exclusion criteria were as follows: patients with incomplete pathological diagnosis data and those who cannot cooperate with MRI examination were excluded.

The article "Diffusion-Weighted Imaging Combined with Perfusion-Weighted Imaging under Segmentation Algorithm in the Diagnosis of Melanoma" was published in 2022. Journal: Contrast Media Mol Imaging.

### 2.2. Instruments and Examination Methods

A 3.0 T MRI examination was performed. The head was scanned with T1WI, T2WI, water suppression, enhanced scanning, and DWI combined with PWI, respectively; and the spinal canal was scanned with T1WI, T2WI, fat suppression, and enhanced scanning. The MRI enhanced scanning contrast agent was gadolinium diethylenetriamine pentaacetic acid (Gd-DTPA), and the intravenous injection dose was 0.1 mmol/kg of weight. The scanning parameters are detailed in Table 1.

### 2.3. Multimodal 3D Image Hybrid Segmentation Algorithm for Intracranial Melanoma

The traditional fuzzy C-means clustering algorithm had the defects of a large amount of calculation and a long running time for large data samples. Therefore, an improved method was proposed to reduce the number of iterations required for the algorithm convergence, and the data sets involved in the iterations were compressed. Therefore, the running time of each iteration process could be reduced, the operation speed of the fuzzy C-means algorithm was improved, and the clustering effect of the algorithm was not affected. The clustering segmentation algorithm of 3D fast fuzzy C-means (FFCM) was carried out by the FFCM, through which the data was divided into *c* categories. For an *P* × *Q* × *W* image, it is assumed that {*g*_*i*_, *i*=1,2,…, *n*; *n*=*P* × *Q* × *W*} was the set of pixel intensity values in the image histogram, {*u*_*j*_, *j*=1,2,…, *c*} was the set of cluster centers, and *μ*_*j*_(*g*_*i*_) was the membership function of g_i_ belonging to category *j*. Thus, the objective function of FFCM is expressed in the following equation:

(1) $$\begin{array}{c} J_{f}=\sum_{j=1}^{c}\sum_{i=1}^{n}{\left[\mu_{j}\left(g_{i}\right)\right]}^{r}{\left\|g_{i}-u_{j}\right\|}^{2}, \end{array}$$

(2) $$\begin{array}{c} \sum_{j=1}^{c}\mu_{j}\left(g_{i}\right)=1,\forall i, \end{array}$$

Together with the equation (2), the FFCM algorithm could be carried out. In the equations, ‖•‖ represented the 2-norm, *r* represented 1-constant>1, which were used to control the fuzzy degree of clustering.

Because the MRI image of intracranial melanoma was extremely complex, a 3D hybrid level set algorithm was applied to integrate the surface and volume information. The zero set of the embedding function *ϕ* was used to represent the active contour *C*={*Y|ϕ*(*Y*)=0}, and the points inside and outside the contour had the positive or negative values. Then the function of minimum need is defined in the following equation:

(3) $$\begin{array}{c} \text{Min}\varepsilon \left(\phi \right)=-\alpha \int_{\Omega }\left(U-\mu \right)W\left(\phi \right)\text{d}\Omega +\beta \int_{\Omega }k|\nabla W\left(\phi \right)|\text{d}\Omega . \end{array}$$

U represented the 3D image to be segmented in the equation (3). *k*=exp(−*c|*∇*U|*^2^) was the surface feature map related to the 3D image gradient, *c* was the control slope, *W*(*ϕ*) was the Heaviside function, Ω was the 3D image area, and *α* and *β* were the predefined weights to balance the two items. Then *μ* stood for the predefined parameter indicating the lower limit of the gray level of the target image.

$\overset{⟶}{Q}$ was defined as the normal vector pointing to the outside of the surface, and then the explicit surface evolution partial differential equation of the active contour could be expressed as the following equation:

(4) $$\begin{array}{c} C_{t}=\alpha \left(U-\mu \right)\overset{⟶}{Q}-\beta \langle \nabla_{k}\overset{⟶}{Q}\rangle +\beta k\kappa \overset{⟶}{Q}. \end{array}$$

In the equation (4), $\overset{⟶}{Q}=-\nabla \phi /|\nabla \phi |$, the curvature *κ*=div(∇*ϕ*/*|*∇*ϕ|*), and 〈·, ·〉 were the inner product. Since only the geometric changes of the curved surface were of interest in the segmentation, it could be observed that all points on the curved surface moved in the normal direction through the equation (4). The first term of the equation (4) represented the transfer item between the expansion motion of the inner surface area and the contraction motion of the outer surface area in the target image. The second term represented the advection item of surface movement in the vector field caused by the gradient *k*, which drew the surface to the boundary of the target object. The third term represented the k-weighted curvature flow of the gradient feature map, meaning that the weak part of the support surface was with a smooth boundary.

The article "Diffusion-Weighted Imaging Combined with Perfusion-Weighted Imaging under Segmentation Algorithm in the Diagnosis of Melanoma" was published in 2022. Journal: Contrast Media Mol Imaging.

In the level set, $C_{t}=\gamma \overset{⟶}{Q}$ and *ϕ*_*t*_=*γ*|∇*ϕ*| represented the same surface change. If *ϕ* was a signed distance function, the derivative of the level set |∇*ϕ*|=1 embedding function over time was described as the following equation:

(5) $$\begin{array}{c} \phi_{t}=\alpha \left(U-\mu \right)+\beta \text{div}\left(k\nabla \phi \right). \end{array}$$

For the process of multimodal 3D image hybrid segmentation algorithm, firstly, the MRI images of T1, T2, and T1ce models were input. Because there was noise in the image itself, the image is preprocessed with median filtering and gray stretching. The gray stretching was applied under the 3D FFCM algorithm, through which partial boundary information could be effectively retained. Then linear fusion was used, and the fused image was for 3D FFCM clustering segmentation. The part with larger gray value in the clustered image was extracted by automatic threshold value, the under-segmented part of intracranial melanoma was then obtained, and finally the mixed level set was used for the segmentation. The flowchart and the main steps of segmentation are shown in Figure 1 and 2.

According to the algorithm flow, the image segmentation steps are shown in Figure 2. Images 2(a)–2(c) represented the original images of FLAIR, T2, and T1C, respectively.  Image 2(d) represented the image obtained after fusion, and images 2(e)–2(g) are processed by FFCM, the automatic threshold, and the mixed level set, respectively.  Image 2(h) was the final image obtained.

## 3. Results

### 3.1. General Data of Patients

Among the 40 patients in this study, 5 cases had the primary lesion in the cerebral meninges, 5 cases had that in the spinal meninges, and 30 cases had intracranial metastatic melanoma. 25 cases and 5 cases had skin and eyeballs as the primary lesion location, respectively.  Figure 3 shows the pictures of melanoma in some patients.

### 3.2. Primary Melanoma

There were 10 cases with primary melanoma in this study. 5 patients were with melanoma in the cerebral meninges and the other 5 with melanoma in the cervical spinal cord. The imaging findings are shown in Table 2 and Figure 4.

From Table 2 and Figure 4, it was found that the primary cerebral meningeal melanoma showed a uniform magnetic signal. A high signal was found on T1WI and T2WI, and a slightly high signal on DWI. As the enhancement scanning was carried out, the lesion area was obviously enhanced, with thickened and enhanced adjacent meningeal nodules and obvious peripheral edema. The PWI suggested that the rCBV of the lesion area of interest was increased. For the primary cervical meningeal melanoma, a typical magnetic signal was found, with a high signal on T1WI and a low signal on T2WI. The adjacent spinal cord suffered from compression; the arachnoid submembrane space was widened; the lesion was obviously enhanced under enhancement scanning, and the dural tail sign of spinal meninges could be observed.

### 3.3. Metastatic Melanoma

There were 30 cases with intracranial metastatic melanoma, including 25 patients with the primary lesion in the skin and 5 patients with the primary lesion in the eyeballs. 20 patients of them were diagnosed with solitary lesion, and 10 patients with multiple lesions. The results of their imaging examinations are shown in Table 3, Figure 5, and6.

From Table 3, Figure 5, and 6, it is observed that most of the patients among the 30 cases with intracranial metastatic melanoma had metastases close to the brain surface, and only a small part of the metastases was located deep. Mild or moderate edema was found around the lesions. The solitary lesions of 20 patients were determined to be of capsule-solid mixed type, with different MRI signals. There were 10 of them who had a low or equally low signal on T1WI and a high or equally high signal on T2WI; and the other 10 patients had mixed signals on T1WI and T2WI. DWI showed high signal or mixed high signal, and significant lesion enhancement was found in all patients under enhancement scanning. For the 10 patients with multiple lesions, their melanomas were all solid, with uniform and typical magnetic signals. Low signal was shown on DWI, and increased rCBV was found on PWI.

The article "Diffusion-Weighted Imaging Combined with Perfusion-Weighted Imaging under Segmentation Algorithm in the Diagnosis of Melanoma" was published in 2022. Journal: Contrast Media Mol Imaging.

### 3.4. Pathological Manifestations

All the patients were diagnosed with melanoma through surgical pathology. The pathological images of some patients are shown in Figure 7.

From Figure 7, most patients had lesions complicated with bleeding. Some patients underwent immunohistochemical test, and the results suggested S-100 protein, malignant melanin-related antigen (HMB45), and Melan-1 were all positive.

## 4. Discussion

The relevant literature stated that primary melanoma of the central nervous system is rare, and it proposed three basic diagnostic conditions, including no melanoma on the skin and eyeballs, no melanoma history of tumor resection, and no melanoma metastasis in internal organs [18]. All the diagnoses of primary melanoma in this study met the above conditions. According to the different locations of the lesions, primary melanoma can be divided into melanoma that diffusely invades the cerebral (spinal) membranes and parenchymal melanoma. The former is more common, mainly because of the widespread existence of melanoma cells in the body, such as the cranial base, brainstem, optic chiasma, dura mater of each lobe of the brain, and spinal membrane [18, 19]. In this study, nodular thickening of the cerebral meninges was observed in cases with primary meningopathy, and obvious enhancement was found during enhanced scanning near the cerebral meninges and sulcus. It was indicated that the meninges were diffusely invaded, and the dural tail sign was only limited to the spinal meninges without any obvious diffusion. It was also suspected that it is because the patients had symptoms of spinal cord compression in the early stages of the rapid growth of the tumor, but due to the timely resection, there was no diffusion to the spinal cord.

MRI shows great differences in the presentation of melanoma, and it can be divided into four types. The first is the melanin type, with T1WI and T2WI with high signal and low signal, respectively. The second is the nonpigmented type, as T1WI and T2WI show equally low signal and equally high signal, respectively. The third is mixed type with the mixed signals; and the fourth is the blood type, with only hemorrhage manifested [20, 21]. When the melanoma is rich in melanin, MRI will be very typical, as T1WI and T2WI showed high signal and low signal, respectively [22]. In this study, the primary spinal meningeal melanoma just belonged to the melanin type. However, the MRI of most melanomas is not typical, and the bleeding and melanin content in the tumor tissues are the main factors in determining the signal of melanoma. Relevant studies have found that to make MRI typical, there must be more than 10% melanocyte content in the tissue. In such a condition, T1WI and T2WI show high signal and low signal, respectively. Peripheral blood vessels are susceptible to melanoma invasion to cause bleeding, but the bleeding signal changes over time, which usually masks the paramagnetic effect of melanin [23, 24]. Among the cases in this study, the signal characteristics of primary meningeal melanoma may be related to the complex tumor signals in the theory.

The article "Diffusion-Weighted Imaging Combined with Perfusion-Weighted Imaging under Segmentation Algorithm in the Diagnosis of Melanoma" was published in 2022. Journal: Contrast Media Mol Imaging.

Metastatic melanoma is more common in the central nervous system, which is the third largest intracranial metastatic tumor, only after that of lung cancer and breast cancer. It may occur in every part of the central nervous system, especially the junctions of the cortex and medulla. The MRI signal performance of it is similar to that of primary melanoma and is also related to bleeding and the content of melanin in tumor tissue [25, 26]. In this study, 30 cases of metastatic melanoma occurred in the brain, most of which were close to the brain surface, and a small portion were located in the deep part of the brain, with various MRI manifestations. 10 cases of multiple metastases with typical signals were all solid ones, and 20 cases of solitary metastases had cystic changes of different degrees. Among the 20 cases, 10 cases were determined to be nonpigmented, with the T1WI and T2WI of low or equally low and high or equally high signal, respectively. The other 10 cases with mixed signals might be related to intracranial bleeding. Melanoma with intracranial metastasis is clinically diagnosed as stage IV, and the survival period is only about 1 year. Therefore, it is particularly important for the accurate identification of the primary melanoma in clinical practice. Intracranial melanoma metastases frequently occur at the junction of the cortex and medulla, mostly with multiple lesions, and primary melanoma mostly occurs in the cerebral meninges. For patients who are highly suspected of having melanoma, their melanoma history should be carefully investigated.

The article "Diffusion-Weighted Imaging Combined with Perfusion-Weighted Imaging under Segmentation Algorithm in the Diagnosis of Melanoma" was published in 2022. Journal: Contrast Media Mol Imaging.

PWI of MRI is applied for the evaluation of the angiogenesis in brain tissues, by measuring cerebral blood volume; while DWI can be used for the analysis of specific tissues. However, the diagnosis of melanoma by PWI combined with DWI is rarely reported at home and abroad [27, 28]. In this study, some patients underwent DWI scanning with the results showing diverse signal manifestations. Primary or solitary metastases showed high or equally high signals of varying degrees, and multiple metastases was shown low signals. Under PWI scanning, rCBV was showed to increase, which suggested the high tumor perfusion. Such results were of some predictive significance for the diagnosis of melanoma.

## 5. Conclusion

In this work, a multimodal 3D image hybrid segmentation algorithm was utilized for observing the MRI findings of melanoma patients. It was discovered that the MRI manifestations of most melanoma patients were complex and diverse, showing different low, high, or mixed signals. DWI combined with PWI examination under the 3D hybrid segmentation algorithm had the advantages of great clarity and accuracy, providing certain value in the diagnosis of melanoma. The disadvantage was that the sample size of this work was small, which needed further supplementation and improvement in the future. This work offered a theoretical reference for the clinical diagnosis and treatment of melanoma.

## Figures and Tables

**Figure 1:** Flowchart of the 3D image hybrid segmentation algorithm.

**Figure 2:** Diagram of the main segmentation steps of intracranial melanoma.

**Figure 3:** Images of melanoma in some patients. (a) Melanoma with raised skin lesions; (b) keratinized melanoma; (c) dyspigmentation; (d) melanoma with irregular borders; (e) 2 or more colors; (f) greater than 5 mm in its diameter.

**Figure 4:** MRI images of primary intracranial melanoma. (A) (B), (C), and (D) : T1WI, T2WI, DWI, and PWI images of cerebral meninges region, respectively. (E) (F) : cervical spinal meninges region, respectively.

**Figure 5:** MRI images of single intracranial metastatic melanoma.

**Figure 6:** MRI images of multiple intracranial metastatic melanomas.

**Figure 7:** Pathological images of melanoma of some patients ( × 200).

**Table 1:** Scanning parameters for the head and spine MRI.

Position	Scanning items	Scanning parameters	Sequence
Head	T1WI	Time of repetition (TR): 2000 ms, time of echo (TE): 9 ms	
	T2WI	TR: 3000 ms, TE: 98 ms	
	Water suppression	TR: 7000 ms, TE: 93 ms Time of inversion (TI): 2500 ms	Fluid attenuated inversion recovery (FLAIR)
	DWI	TR: 5000 ms, TE: 90 ms	
	PWI	TR: 1500 ms, TE: 60 ms Slice thickness: 5 mm	

Spinal canal	T1WI	TR: 420 ms, TE: 9 ms	
	T2WI	TR: 3000 ms, TE: 113 ms	
	Fat suppression	TR: 330 ms, TE: 41 ms	Turbo inversion recovery magnitude (TIRM)
		TI: 220 ms	
		Slice thickness: 3 mm	

The article "Diffusion-Weighted Imaging Combined with Perfusion-Weighted Imaging under Segmentation Algorithm in the Diagnosis of Melanoma" was published in 2022. Journal: Contrast Media Mol Imaging.

**Table 2:** Imaging results of primary melanoma.

		High signal	Slightly high signal	Low signal
Cerebral meninges	T1WI	√		
	T2WI	√		
	DWI		√	
	PWI	The relative cerebral blood volume (rCBV) of the lesion area of interest was increased.		

Cervical spinal meninges	T1WI	√		
	T2WI			√

**Table 3:** Imaging results of intracranial metastatic melanoma.

		High or equally high signal	Low or equally low signal	Mixed signal	Low signal
Solitary	T1WI		√	√	
	T2WI	√			
	DWI	All equally high signals or mixed high signal			

Multiple	DWI				√
	PWI	Increasing rCBV on the solid parts of lesions			

## Data Availability

The data used to support the findings of this study are available from the corresponding author upon request.

## References

[1] Cabrera R., Recule F. (2018). Unusual clinical presentations of malignant melanoma: a review of clinical and histologic features with special emphasis on dermatoscopic findings. *American Journal of Clinical Dermatology*.

[2] Fujimoto M., Matsuzaki I., Nishitsuji K. (2020). Adipophilin expression in cutaneous malignant melanoma is associated with high proliferation and poor clinical prognosis. *Laboratory Investigation*.

[3] Mastoraki A., Schizas D., Giannakodimos I. (2020). Malignant melanoma of the breast: controversies in the diagnosis and therapeutic management of a rare nosologic entity. *International Journal of Dermatology*.

[4] Yang N., Lu J., Lu Y., Guo J., Wang H. (2019). Primary malignant melanotic melanoma and hypomelanotic melanoma of the female urethra: case series and a review of the literature in China. *Melanoma Research*.

[5] Harrington E., Clyne B., Wesseling N. (2017). Diagnosing malignant melanoma in ambulatory care: a systematic review of clinical prediction rules. *BMJ Open*.

[6] Shao J.-W., Yin J.-H., Xiang S.-T., He Q., Zhou H., Su W. (2020). CT and MRI findings in relapsing primary malignant melanoma of the lacrimal sac: a case report and brief literature review. *BMC Ophthalmology*.

[7] Kawaguchi M., Kato H., Tomita H. (2020). MR imaging findings for differentiating cutaneous malignant melanoma from squamous cell carcinoma. *European Journal of Radiology*.

[8] Francis J. H., Catalanotti F., Landa J., Barker C. A., Shoushtari A. N., Abramson D. H. (2019). Hepatic abnormalities identified by staging MRI and accuracy of MRI of patients with uveal melanoma. *British Journal of Ophthalmology*.

[9] Jaarsma-Coes M. G., Goncalves Ferreira T. A., van Haren G. R., Marinkovic M., Beenakker J.-W. M. (2019). MRI enables accurate diagnosis and follow-up in uveal melanoma patients after vitrectomy. *Melanoma Research*.

The article "Diffusion-Weighted Imaging Combined with Perfusion-Weighted Imaging under Segmentation Algorithm in the Diagnosis of Melanoma" was published in 2022. Journal: Contrast Media Mol Imaging.

[10] Mosavi F., Ullenhag G., Ahlström H. (2013). Whole-body MRI including diffusion-weighted imaging compared to CT for staging of malignant melanoma. *Upsala Journal of Medical Sciences*.

[11] Gumeler E., Parlak S., Yazici G., Karabulut E., Kiratli H., Oguz K. K. (2021). Single shot echo planar imaging (ssEPI) vs single shot turbo spin echo (ssTSE) DWI of the orbit in patients with ocular melanoma. *British Journal of Radiology*.

[12] Young G. S., Setayesh K. (2009). Spin-echo echo-planar perfusion MR imaging in the differential diagnosis of solitary enhancing brain lesions: distinguishing solitary metastases from primary glioma. *American Journal of Neuroradiology*.

[13] Hu M., Zhong Y., Xie S., Lv H., Lv Z. (2021). Fuzzy system based medical image processing for brain disease prediction. *Frontiers in Neuroscience*.

[14] Fan N., Yuan S., Du P. (2020). Design of a robot-assisted system for transforaminal percutaneous endoscopic lumbar surgeries: study protocol. *Journal of Orthopaedic Surgery and Research*.

[15] Xie S., Yu Z., Lv Z. (2021). Multi-disease prediction based on deep learning: a survey. *Computer Modeling in Engineering and Sciences*.

[16] Jaarsma-Coes M. G., Ferreira T. A., Luyten G. P. M., Beenakker J. W. M. (2019). Reaction on “Ocular ultrasound versus MRI in the detection of extrascleral extension in a patient with choroidal melanoma”. *BMC Ophthalmology*.

[17] Lv Z., Qiao L. (2020). Analysis of healthcare big data. *Future Generation Computer Systems*.

[18] Sladden M. J., Nieweg O. E., Howle J., Coventry B. J., Thompson J. F. (2018). Updated evidence based clinical practice guidelines for the diagnosis and management of melanoma: definitive excision margins for primary cutaneous melanoma. *Medical Journal of Australia*.

[19] Chen D., Wawrzynski P., Lv Z. (2020). Cyber security in smart cities: a review of deep learning-based applications and case studies. *Sustainable Cities and Society*.

[20] Piscioli F., Pusiol T., Roncati L. (2016). Nowadays a histological sub-typing of thin melanoma is demanded for a proper patient management. *Journal of Plastic, Reconstructive & Aesthetic Surgery*.

[21] Zeng Y., Zeng Y., Yin H. (2021). Exploration of the immune cell infiltration-related gene signature in the prognosis of melanoma. *Aging (Albany NY)*.

[22] Su Y., Xu X., Zuo P. (2020). Value of MR-based radiomics in differentiating uveal melanoma from other intraocular masses in adults. *European Journal of Radiology*.

[23] Kim Y.-K., Choi J. W., Kim H.-J. (2018). Melanoma of the sinonasal tract: value of a septate pattern on precontrast T1-weighted MR imaging. *American Journal of Neuroradiology*.

The article "Diffusion-Weighted Imaging Combined with Perfusion-Weighted Imaging under Segmentation Algorithm in the Diagnosis of Melanoma" was published in 2022. Journal: Contrast Media Mol Imaging.

[24] Liu J., Chen J., Zha Y., Huang Y., Zeng F. (2021 Jul). Magnetic resonance imaging (MRI) differential diagnosis of meningiomas using ANOVA. *Contrast Media and Molecular Imaging*.

[25] Tang S., Zuo J., Zhang H., Wu Z., Liang B. (2020). Spinal metastatic melanoma with unknown primary lesions presenting as radiculopathy: case report and literature review. *World Neurosurgery*.

[26] LoRusso P. M., Schalper K., Sosman J. (2020). Targeted therapy and immunotherapy: emerging biomarkers in metastatic melanoma. *Pigment Cell & Melanoma Research*.

[27] Askaner K., Rydelius A., Engelholm S. (2019). Differentiation between glioblastomas and brain metastases and regarding their primary site of malignancy using dynamic susceptibility contrast MRI at 3T. *Journal of Neuroradiology*.

[28] McDonald M. A., Sanghvi P., Bykowski J., Daniels G. A. (2018). Unmasking of intracranial metastatic melanoma during ipilimumab/nivolumab therapy: case report and literature review. *BMC Cancer*.

